# Application and Research of Computer Intelligent Technology in Modern Agricultural Machinery Equipment

This article has been retracted.

**DOI:** 10.1155/2022/9978167

**Published:** 2022-08-09

**Authors:** Hongyu Zhou, Jinqi Liu, Fan Huang

**Affiliations:** ^1^Hubei University of Technology, Wuhan 430068, China; ^2^Hubei Packaging Equipment Engineering Technology Research Center, Wuhan 430068, China

## Abstract

Every country, including China, is deeply concerned and interested in the topic of agricultural machinery automation. The world's population is growing at an astronomical rate, and as a result, the need of food is also growing at an astronomical rate. Farmers are forced to apply more toxic pesticides since traditional methods are not up to the task of meeting the rising demand. This has a major impact on agricultural practices, and in the long run, the land becomes barren and unproductive. Intelligent technologies such as Internet of Things, wireless communication, and machine learning can help with crop disease and pesticide storage management, as well as water management and irrigation. In this paper, we design and analyze an intelligent system that automatically predicts the agricultural land features for irrigation purpose. Initially, the dataset is collected and preprocessed using normalization. The features are extracted using principal component analysis (PCA). For automatic prediction by the equipment, we propose heterogeneous fuzzy-based artificial neural network (HF-ANN) with genetic quantum spider monkey optimization (GQ-SMO) algorithm. Analyses and comparisons are made between the proposed approach and current methodologies. The findings indicate the effectiveness of the proposed system.

## 1. Introduction

Agriculture had played a significant part in a global economy in recent years. It is inevitable that as the population grows, urbanization will lead to a progressive decrease in the area of farmed land, which will put further strain on the agricultural system. Agricultural food production systems that are both efficient and safe are in high demand. The growth of high-quality and high-yield agricultural will be aided if traditional agricultural management approaches are supplemented with novel sensing and driving technologies and better information and communication technology. Computer vision inspection technologies have grown in importance in agricultural operations over the last few decades and have seen a rise in their utilization. Automated agricultural production management systems based on computer visual algorithms are becoming more and more popular in the agricultural sector (Tian et al. [1] and Mody and Bhoosreddy [2]). The next step of agricultural production is called “intelligent agriculture.” Accomplishment of the following aims can be achieved by fully employing contemporary information technology (including perception, connectivity, and intelligent techniques): farm products have a strong competitive advantage and are well protected by the environment. Rural regions are harmonious, and the use of rural energy is efficient. There have been a number of policies and demonstration projects put in place by China in this regard. The Opinions on Accelerating a Transformation of Agriculture Modes suggested that Agri-IoT mature and repeatable application modes be promoted, precision production modes be established, and energetic regional pilot programs for Agri-IoT be executed (Hu et al. [3]).

Modern information technologies including the Internet of Things, big information, artificial intelligence, and human interactions are being used to a range of agricultural operations as part of a new tendency in food production termed “intelligent agriculture.” Computer-assisted agricultural production (CAAP) is expected to boost productivity, reduce costs, and improve the ecosystem through the implementation of IA (Shi et al. [4] and Garg [5]). The combination of modern manufacturing and information technology is a key development direction for contemporary manufacturing technologies. “Industrial Internet” (deep integration of IT and manufacturing) and “Sector 4.0” (promotion of intelligence manufacturing) have all been introduced in the last few years, and one of the ultimate aims of a manufacturing industry is now Made in China 2025. Information technology is essential to advancing this intelligent transformations of traditional manufacturing, and it is beginning to permeate all facets for mechanical machining operations in particular (Lv et al. [6] and Shahabaz and Afzal [7]).

Traditional farming methods are becoming more and more automated as the population grows and the need for food rises, leading to a significant agricultural advancement. Today, a wide range of machines and equipment are available for a variety of agricultural activities, including product harvesting, where farmers have a significant challenge in selecting the optimum machine based on efficiency and other variables.  Figure 1 depicts the agricultural machinery and technologies. Olive picking is a good illustration of this. In this regard, they look at six machines and equipment as options, as well as some beneficial elements as criteria for making a pick. For harvesters, combs can be harvested with a number of tools such as handheld harvesters, straddle and umbrella shaker, and tractor-mounted harvesters (Hafezalkotob et al. [8]).

Hence, application and research of computer intelligent technology in modern agricultural machinery equipment are investigated in this article. The further portion of the paper is structured as shown: Section 2 provides the associated literature and the problem statement. The flow of the proposed work is explained in Section . Section examines and compares the proposed method's behavior to that of traditional approaches. Finally, Section brings the paper's overarching theme to a close.

## 2. Related Works

The use of machine learning in agriculture is provided by the authors. Organic carbon and moisture content in the soil, agricultural yield prediction, disease and weed identifications in crops, and species identification are all areas of study. Classification of crop photos based on machine learning (ML) and computer vision is examined to monitor crop quality and yield evaluation (Sharma et al. [9]). Idoje et al. [10] proposed that there is a need for more research on the difficulties of applying smart technology to farming, and this study helps fill that gap by outlining concerns raised already by the existing framework for smart agriculture. Orishev et al. [11] investigates the potential benefits and projected future development opportunities for computer intelligence technology in agriculture. According to a survey of recent publications on the evolution of intelligent technologies in agriculture, it is obvious that intelligence technologies are widely used in the agricultural industry. Each technique's potential for specialized application is examined in [12] and [13], which provides an overview for instructive examples in various agricultural fields using statistical machine learning approaches now being used in machine vision systems. A worldwide perspective is taken on the usage of machine learning, computer vision, and deep learning in various situations and applications. It is becoming increasingly fashionable to employ computer vision and artificial intelligence to grow food responsibly for the future (Kakani et al. [14]). Pathan et al. [15] reviewed some of the agricultural intelligence applications that include precision farming, disease forecasting, and crop phenotyping. A variety of tools, such as machine learnings, artificial neural networks, convolutional neural networks, wireless communications, robotic devices, the Internet of Things, genetic algorithms, fuzzy logic, and computer vision, will be used to analyze these applications. Agriculture technology applications and research activities will be reviewed in this article, focusing on the evolution of these technologies in the context of “smart farming” (Charania and Li [16] and Salihu and Zayyanu [17]).

Agriculturists will appreciate this writer's Internet of Things (IoT) platform-based smart controls and monitoring methods for agricultural machinery. Accuracy is critical to irrigation systems since they can operate even when the energy source is disrupted (Rajan et al. [18]). From a standpoint of organizational function, this article intends to explain each structural part's information technologies function as well as its relationships with other technologies in order to enhance computer intelligent agriculture (Deng [19] and Ahmed and Aatiqa [20]). Sustainable and intelligent precision agriculture is the subject of the studies included in this special section (Shu et al. [21]). Industrial revolutions have taken place three times during the course of human history. Everything from labor-intensive farming and automated manufacturing to big scale fine-grained industrial agriculture is radically altered by each industrial revolution.

### 2.1. Problem Statement

Due to a lack of use of modern technologies, agricultural activities in China have remained mostly basic during the previous few decades. Tractors, harvesters, planters, and other agricultural gear are too expensive for the typical China farmer. Obtaining long-term funding to expand their farms, invest in productive assets, or acquire supplies is a difficult task. Agricultural financing has suffered serious setbacks for several years as a result of a number of impeding factors, including low agricultural productive output, a lack of capital and inaccessibility to credit establishments, a lack of adequate inputs and storage areas, an unfavorable and nonenabling environments, weak agricultural extension, and outdated sectoral infrastructure. However, there is a paucity of research on the impact of agricultural technical (equipment) funding on China's productivity and industrialization, despite the abundance of literature on these topics.

## 3. Proposed Work

This part explains the flow of the suggested methodology. The schematic representation of the suggested technique includes the processes like analyzing the information collection from soil, feed information to the system, data preprocessing using normalization, feature extraction using principle component analyses, prediction using heterogeneous fuzzy-based artificial neutral network, genetic quantum spider monkey optimization, and performance analyses in application and research of computer intelligent technology in modern agricultural machinery equipment. The schematic representation of the suggested technique is depicted in Figure 2.

### 3.1. Information Collection from Soil

While China possesses 133.39 million acres (ha) of arable land, this is less than half of the country's population. Particularly, big portions of the country's agricultural land are in Heilongjiang, Inner Mongolia, Henan, Hebei, and Shandong. In Shanghai, Beijing, and Tianjin, the total arable area is less than 1% in China's entire arable land. It was determined that there were 31 provinces/municipalities on China's mainland that could be categorized into seven primary areas because of data limitations (shown in Table 1) (Han and Li [22]).

### 3.2. Feed Information to the System

A data feed can stream constantly or be given on demand. Data feed makes it feasible to have fresh material or updates provided to a system or mobile devices as soon as it is released. The same methods were also used to give data to other apps.

### 3.3. Data Preprocessing Using Normalization

Normalization is a preprocessing technique used to enhance the RCAIL dataset. Normalized values of an attribute in a dataset fall within a predetermined range, such as 0.0 to 1.0, which is specified in the dataset. Normalization smoothes and normalizes data before modeling. To make it easier to put the concept into practice, common mathematical transformations are used. There are a number of ways to normalize data, such as “min-max normalization,” “*z*-score normalization,” and “decimal scaling normalization.”

#### 3.3.1. *Z*-Score Normalization

To accomplish *Z*-score normalization, also called zero normalization, the mean and standard deviation for each characteristic in a training set are obtained and divided by a number of variables in a training dataset. The mean and standard deviation are determined for each attribute. The transformation to be done is specified in the general formula:

(1) $$\begin{array}{c} c=\frac{\left(c-\mu \right)}{\sigma }, \end{array}$$

where the property c's average is *μ* and its standard deviation is *σ*. All of the features in the dataset are normalized using the *z*-score process before training can begin. After a set of training data has been computed, it is critical to maintain the standard deviation and mean for each feature so that they may be utilized as weights in the system's design.

#### 3.3.2. Min-Max Normalization

This equation is used in min-max normalization to normalize features in the interval [0, 1].

(2) $$\begin{array}{c} u^{\prime }=\frac{u-\min_{P}}{\max_{P}-\min_{P}}. \end{array}$$

min_*p*_ and max_*p*_ are the values of a feature A's minimal and maximum values. *u* and *u*^,^ indicate the attribute *P* original and normalized values, respectively. The preceding equation shows that the maximum and minimum feature values are mapped as 1 and 0 accordingly, as can be seen from the equation.

### 3.4. Feature Extraction Using Principle Component Analysis (PCA)

The PCA has been widely used in a number of fields because to its simplicity and ease of understanding, as well as the fact that it has no parameter constraints. Using PCA, m-dimensional variables may be reduced to l-dimensional features. There are new orthogonal l-dimensional elements formed from the m-dimensional features, known as fundamental components. The PCA removes data duplication while sacrificing the least amount of information possible in order to achieve its dimension reduction goals.

The steps of the PCA are divided into the following segments:

Step 1: the PCA's stages are divided into the following categories, where *h* =  *h*_1_, *h*_2_,…, *h*_*J*_.
  (3) $$\begin{array}{c} \propto =\frac{1}{j}\sum_{n=1}^{j}h_{a}, \end{array}$$
  where *j* indicates the selection chosen in example *n* = 1, and…, *j*.
Step 2: covariance matrix for the example set is calculated using the sample mean.
  (4) $$\begin{array}{c} P=\frac{1}{j}\sum_{a=1}^{j}\left(h_{a}-\propto \right){\left(h_{a}-\propto \right)}^{o}. \end{array}$$
  where *P* is the covariance matrix of the sample set.
Step 3: the sample covariance matrix's feature values and feature vectors must be determined.
  (5) $$\begin{array}{c} P=K.\Sigma .K^{T},\\ \Sigma =\text{diag}\left(\lambda_{1},\lambda_{2,\ldots ,}\lambda_{s}\right)\lambda_{1}\geq \lambda_{2}\geq \ldots \geq \lambda_{s}\geq 0,\\ K=\left[k_{1},k_{2,\ldots ,}k_{s}\right]. \end{array}$$
P is the down-ordered structured diagonal matrices of *m* covariance matrices quality values, covariance matrices attribute values *λ*_*j*_ are shown below, and attribute vector *k*_*j*_ of feature value *λ*_*j*_ is used to construct quality matrix *K*, *i* = 1,…, *s*.
Step 4: using the feature ratings and feature vectors derived from first l-row primary elements, for the first l-row main items, we compute the cumulative deviation pension contribution:
  (6) $$\begin{array}{c} \theta =\frac{\sum_{j=1}^{l}\lambda_{j}}{\sum_{i=1}^{n}\lambda_{j}}. \end{array}$$
  where *θ*indicates the cumulative variation contribution rate of former l-row primary components and is frequently more than or equal to 0.9. In principle, the element should be as high. The element must be carefully selected in light of a specific issue to be handled from a practical perspective. The specifics of restated initial selections set of the *k*-row major components can be ascertained if the value is suitably chosen.
Step 5: reduce the dimensions using the *q*-row feature vector that was just collected.
  (7) $$\begin{array}{c} A=K_{l},\\ X=A.Y. \end{array}$$

For the initial *k*-row quality importance (*l* ≤ *n*), P is a characteristic matrices derived from the matching quality vectors. The first *k* rows of a feature matrix, *Q*_*l*_, must be filled up. *L*-dimensional data are represented by the symbol *Y*. As a result, the unbent data may be transformed from *m*-dimensional (*Y*) into linear (*X*) dimensions in order to achieve linearization.

### 3.5. Prediction Using the Heterogeneous Fuzzy-Based Artificial Neural Network

Prediction intervals using fuzzy and artificial neural network models with heterogeneous properties are developed in this part. When used for recognition, an artificial neural network (ANN) often lacks the flexibility to be tailored to a specific job within an acceptable amount of time. Heterogeneous fuzzy modeling, in contrast, necessitates a strategy to learning from experiences (i.e., data acquired in advance) in order to fuse the judgments made by the many variables. Sixth-generation systems research is divided into three areas: ANNs, heterogeneous fuzzy logic, and genetic systems. There are several applications for the fuzzy ANNs, which use a heterogeneous fuzzy model, and each has its own set of benefits and drawbacks. For the discipline to move further, understanding how ANNs and fuzzy modeling interact is critical.

The classic heterogeneous fuzzy system, as described above, relies on the expertise of subject matter experts. That being said, it does not appear to be particularly impartial. Aside from that, finding reliable information and qualified human specialists is quite tough. A new and promising technique to improving the performance of a heterogeneous fuzzy system has been demonstrated using ANN's learning algorithm. A feedforward neural network (ANN) was incorporated into fuzzy inference by the researcher. An ANN represents each rule, but a single ANN represents all membership functions. Partitioning the inference rules, identifying IF components, and identifying THEN components are the three main components of the algorithm. There are distinct artificial neural networks for each rule and each membership function; therefore, they are all trained individually. As a result, the variables cannot be modified at the same time. The fuzzy neural networks (FNNs) referred to in this article are only suitable for numerical data. But even so, specialists' knowledge tends to be of the fuzziness variety. Because of this, several scientists are trying to solve this issue. Using fuzzy if–then rules, artificial neural networks may learn from both numerical input and expert knowledge.

(8) $$\begin{array}{c} \overset{¯}{X}\left(x\right)=\left(\bar{Y}+\bar{Z}\right)\left(x\right),\\ \bar{X}\left(x\right)=\max\left\{\bar{Y}\left(y\right)\Lambda \bar{Z}\left(z\right)|x=y+z\;\right\},\\ \bar{X}\left(x\right)=\max\left\{\bar{Y}\left(y\right)\Lambda \bar{Z}\left(z\right)|x=y\cdot z\;\right\},\\ \bar{X}\left(x\right)=\left(\bar{Y\;}\cdot \bar{Z}\right)\left(x\right),\\ \bar{X}\left(x\right)=\max\left\{\bar{\text{Net}}\left(y\right)|x=f\left(y\right)\;\right\}. \end{array}$$

To fine-tune a proposed FNN's input, weights, and output vector from multilayer feedforward neural networks, fuzzy numbers must be combined, multiplied, and mapped in nonlinear ways.

### 3.6. Genetic Quantum Spider Monkey Optimization

Spider monkeys' behavior is mimicked by a quantum spider monkey optimization (QSMO) technique, which uses the fission-fusion social structures (FFSS). This algorithm was inspired by spider monkeys' foraging habits. In South American nations, spider monkeys are an indigenous species. Spider monkeys' social behavior is already predicated on intelligence, thanks to the species' self-organizing foraging habit. In addition, they create subgroups in the monkey community to divide the members of the group in order to decrease independent foraging among themselves. The fitter a monkey becomes, the closer it gets to its meal. Other spider monkeys are encouraged to approach food as a result of their proximity to it. Swarm nature means that QSMO algorithm typically ends up at a fixed point, even if its equilibrium states tend to alternate between diversity and intensification.

Cooperative iterative processes based on trial and error are used in the spider monkey optimization method. In this way, the global optimum may be achieved with the smallest number of iterations possible. Local leaders (LLs) and global leaders (GLs) are used in the QSMO algorithm. The suggested QSMO approach begins with the quantum coding of a randomly distributed spider monkey populations *P* to a D-dimensional vector SM_*ii*_  = 1, 2,…, *P*, and the *SM*_*ii*_  = 1, 2,…, *P* vectors are created. Because of this, *D* and SM_*i*_ are the variables in the optimization problems and SM_*i*_ is the population's *I* th spider monkey. Using the procedure, all particles' positions are changed after the evaluation of their fitness and that of the local leader (LL).

### 3.7. Performance Analysis

The overall behavior of the recommended framework is discussed in this section. The comparison of metrics such as maximum absolute errors, normalized mean absolute errors, root mean square error, normalized root mean square error, and prediction accuracy for current and new approaches is shown in Figures 3–7. Support vector machines, multiple regression, random forest, and deep neural networks are some of the methods used.

Figure 3 represents the maximum absolute errors with proposed and existing approaches. The proposed method of heterogeneous fuzzy-dependent artificial neural network exhibits low maximum absolute errors when compared to current methodologies such as support vector machines (SVMs), multiple regression, random forest (RF), and deep neural networks.

Figure 4 represents the normalized mean absolute errors with proposed and existing approaches. Figure 4 shows that the proposed method of heterogeneous fuzzy-based artificial neural network has low normalized mean absolute errors, when compared to the existing methods such as support vector machine, multiple linear regression, random forest, and deep neural network.

Figure 5 represents the root mean square errors with proposed and existing approaches. Figure 5 shows that the proposed method of heterogeneous fuzzy-based artificial neural network has low root mean square errors, when compared to the existing methods such as support vector machine, multiple linear regression, random forest, and deep neural network.

Figure 6 represents the normalized root mean square errors with proposed and existing approaches. Figure 3 shows that the proposed method of heterogeneous fuzzy-based artificial neural network has low normalized root mean square errors, when compared to the existing methods such as support vector machine (SVM), multiple linear regression (MLR), random forest (RF), and deep neural network (DNN).

Figure 7 represents the prediction accuracy with proposed and existing approaches. Figure 3 shows that the proposed method of heterogeneous fuzzy-based artificial neural network has high prediction accuracy, when compared to the existing methods such as support vector machine, multiple linear regression, random forest, and deep neural network.

## 4. Discussion

In this section, we evaluate the efficacy of our suggested approach using the performance indicator indicated before. As per Table 1, the datasets are gathered for China's regional divisions. The preprocessing stage is carried out to standardize/balance the given datasets through normalization techniques. Our proposed technique is performed and also matched with other standard techniques: SVM (Taghizadeh et al. [23]), MLR (Knoll et al. [24]), RF (Talukdar et al. [25]), and DNN (Liakos et al. [26]). Large datasets are not suited for the SVM method. SVM does not function well when a dataset contains extra noise, including as overlapping target classes. When the number of variables of each data point exceeds the amount of training data samples, an SVM may underperform. In multiple linear regression, the drawbacks of the quality of the data are almost always the deciding factor in whether or not to utilize a multiple regression model. There are two examples of this: the use of inadequate data and the erroneous conclusion that a connection is causal. Random forest's capacity to manage large numbers of trees makes it unsuitable for real-time forecasts. These algorithms are very simple to learn, but they require a long time to forecast after they had been taught. It takes a large amount of data to perform better than other tactics. Training is highly costly due to the sophisticated data models. The utilization of hundreds of expensive GPUs is required for deep neural networks. This increases the cost to customers.

Figure 3 depicts the comparison of maximum absolute errors with proposed and existing techniques regarding the given financial collections. In this graph, the *x*-axis denotes financial datasets and the *y*-axis denotes maximum absolute errors. In Figure 3, the existing methods of support vector machine have 63%, multiple linear regression has 70%, random forest has 65%, deep neural network has 74%, and the proposed method of heterogeneous fuzzy-based artificial neural network has 58%, so when compared to the existing methods the proposed method has low maximum absolute errors.

Figure 4 depicts the comparison of normalized mean absolute errors with proposed and existing techniques regarding the given financial collections. In this graph, the *x*-axis denotes financial datasets and the *y*-axis denotes normalized mean absolute errors. In Figure 4, the existing methods of support vector machine have 58%, multiple linear regression has 62%, random forest has 70%, deep neural network has 64%, and the proposed method of heterogeneous fuzzy-based artificial neural network has 55%, so when compared to the existing methods the proposed method has low normalized mean absolute errors.

Figure 5 depicts the comparison of root mean square errors with proposed and existing techniques regarding the given financial collections. In this graph, the *x*-axis denotes financial datasets and the *y*-axis denotes root mean square errors. In Figure 5, the existing methods of support vector machine have 64%, multiple linear regression has 58%, random forest has 68%, deep neural network has 61%, and the proposed method of heterogeneous fuzzy-based artificial neural network has 50%, so when compared to the existing methods the proposed method has low root mean square errors.

Figure 6 depicts the comparison of normalized root mean square errors with proposed and existing techniques regarding the given financial collections. In this graph, the *x*-axis denotes financial datasets and the *y*-axis denotes normalized root mean square errors. In Figure 6, the existing methods of support vector machine have 58%, multiple linear regression has 62%, random forest has 64%, deep neural network has 55%, and the proposed method of heterogeneous fuzzy-based artificial neural network has 40%, so when compared to the existing methods the proposed method has low root normalized root mean square errors.

Figure 7 displays the comparison of prediction accuracy for suggested and current strategies with reference to the provided financial collection. In this graph, the *x*-axis denotes financial datasets and the *y*-axis denotes prediction accuracy. In Figure 7, the existing methods of support vector machine have 58%, multiple linear regression has 52%, random forest has 45%, deep neural network has 55%, and the proposed method of heterogeneous fuzzy-based artificial neural network has 65%, so when compared to the existing methods the proposed method has low root prediction accuracy.

## 5. Conclusion

A potential agricultural automation use of computer intelligent technology was assessed based on the current state of affairs. First, since technology continues to advance, a large-scale dataset is needed in order to realize technology's adaptability and coordination. In addition, new technologies and problems will continue to arise in the future. Second, as agricultural automation progresses, more disciplines will be integrated, increasing the demand for specialists in terms of both quality and quantity. It will be difficult to ensure the accuracy and robustness of associated technologies in many complicated conditions because of agricultural production management's environmental complexity.

Our conclusion is that computer intelligent technology will be better suited to agriculture because it is a new and emerging technology. Computing power derived from large-scale datasets and used to computer visual intelligence will be increasingly common in agricultural production management in the future. Artificial intelligence algorithms and computer intelligent technologies can increase the economic, general, coordination, and robustness of agricultural automation system. Agricultural automations equipment and systems will become more intelligent when cutting-edge technology such as deep learning and spectrum analysis is applied. As computer intelligent technology advances, agricultural productivity and quality will be enhanced, and farmers will be able to rely on the technology's suggestions and insights to help them make better decisions and take better action. This will also aid in the rapid and complete development of agricultural machinery equipment. The limitation of the present study is computer-assisted farming must have an unlimited or constant Internet connection. Due to huge crop production in developing countries, this farming practice is impractical especially in rural areas. Agricultural production management in the future will increasingly rely on computer intelligent technology based on large-scale datasets, which will be utilized to tackle existing agricultural challenges. The use of computer intelligent technology and AI techniques will increase agricultural automation systems' economic, general, coordinated, and resilient performance. Agricultural automation equipment and systems will become more intelligent when cutting-edge technologies such as deep learning and spectrum analysis are used. Farmers will be able to make better decisions and take action with the use of computer vision technology, which is expected to boost agricultural productivity in the future and promote the quick and comprehensive growth of agricultural automation.

## Figures and Tables

**Figure 1:** Agricultural machinery and technology.

**Figure 2:** Schematic representation of the suggested methodology.

**Figure 3:** Maximum absolute errors of the proposed and existing methodology.

**Figure 4:** Normalized mean absolute errors of the proposed and existing methodology.

**Figure 5:** Root mean square errors of the proposed and existing methodology.

**Figure 6:** Normalized root mean square errors of the proposed and existing methodology.

**Figure 7:** Prediction accuracy of the proposed and existing methodology.

**Algorithm 1:** The QSMO algorithm.

**Table 1:** China's regional divisions.

No.	Category	Province/municipality
1	East China	Shanghai, Jiangsu, Zhejiang, Anhui, Fujian, Jiangxi, Shandong
2	Central China	Henan, Hubei, Hunan
3	North China	Beijing, Tianjin, Hebei, Shanxi, Inner Mongolia
4	Northwest China	Shaanxi, Gansu, Qinghai, Ningxia, Xinjiang
5	Southwest China	Chongqing, Sichuan, Guizhou, Yunnan, Tibet
6	Northeast China	Liaoning, Jilin, Heilongjiang
7	South China	Guangdong, Guangxi, Hainan

## Data Availability

The data used to support the findings of this study are available from the corresponding author upon request.

## References

[1] Tian H., Wang T., Liu Y., Qiao X., Li Y. (2020). Computer vision technology in agricultural automation -a review. *Information Processing in Agriculture*.

[2] Mody R. N., Bhoosreddy A. R. (1995). Multiple odontogenic keratocysts: a case report. *Annals of Dentistry*.

[3] Hu X., Sun L., Zhou Y., Ruan J. (2020). Review of operational management in intelligent agriculture based on the internet of things. *Frontiers of Engineering Management*.

[4] Shi L., Shi G., Qiu H. (2018). General review of intelligent agriculture development in China. *China Agricultural Economic Review*.

[5] Garg H. (2020). Digital twin technology: revolutionary to improve personalized healthcare. *Science Progress and Research (SPR) 1*.

[6] Lv L., Deng Z., Liu T., Li Z., Liu W. (2020). Intelligent technology in grinding process driven by data: a review. *Journal of Manufacturing Processes*.

[7] Shahabaz A., Afzal M. (2021). Implementation of high dose rate brachytherapy in cancer treatment. *Science Progress and Research*.

[8] Hafezalkotob A., Hami-Dindar A., Rabie N., Hafezalkotob A. (2018). A decision support system for agricultural machines and equipment selection: a case study on olive harvester machines. *Computers and Electronics in Agriculture*.

[9] Sharma A., Jain A., Gupta P., Chowdary V. (2020). Machine learning applications for precision agriculture: a comprehensive review. *IEEE Access*.

[10] Idoje G., Dagiuklas T., Iqbal M. (2021). Survey for smart farming technologies: challenges and issues. *Computers & Electrical Engineering*.

[11] Orishev A. B., Mamedov A. A., Sycheva I. N., Sherstyuk M. V. (2020). Promising intelligent technologies for agricultural development. *intelligent technologies in agriculture*.

[12] Rehman T. U., Mahmud M. S., Chang Y. K., Jin J., Shin J. (2019). Current and future applications of statistical machine learning algorithms for agricultural machine vision systems. *Computers and Electronics in Agriculture*.

[13] Li Z. (2022). *Treatment And Technology Of Domestic Sewage For Improvement Of Rural Environment In China-Jiangsu: A Research, SPR*.

[14] Kakani V., Nguyen V. H., Kumar B. P., Kim H., Pasupuleti V. R. (2020). A critical review on computer vision and artificial intelligence in food industry. *Journal of Agriculture and Food Research*.

[15] Pathan M., Patel N., Yagnik H., Shah M. (2020). Artificial cognition for applications in smart agriculture: a comprehensive review. *Artificial Intelligence in Agriculture*.

[16] Charania I., Li X. (2020). Smart farming: agriculture’s shift from a labor intensive to technology native industry. *Internet of Things*.

[17] Salihu S. O., Zayyanu I (2022). Assessment of physicochemical parameters and Organochlorine pesticide residues in selected vegetable farmlands soil in Zamfara State, Nigeria. *Science Progress and Research (SPR)*.

[18] Rajan V. K., Sengolrajan T., Arul P., Raghavendran P. S. (2021). Eco friendly modern agriculture machinery control and monitoring with IoT. *Nveo-Natural Volatiles & Essential Oils Journal Nveo*.

[19] Deng T. (2021). Study of the system construction and development path of intelligent agriculture in China. *Cultures of Science*.

[20] Ahmed B., Aatiqa A. (2020). Usage of traditional Chinese medicine, western medicine and integrated Chinese-western medicine for the treatment of allergic rhinitis. *Official Journal of the Zhende Research Group 1*.

[21] Shu L., Hancke G. P., Abu-Mahfouz A. M. (2021). Guest editorial: sustainable and intelligent precision agriculture. *IEEE Transactions on Industrial Informatics*.

[22] Han M., Li S. (2021). Transfer patterns and drivers of embodied agricultural land within China: based on multi-regional decomposition analysis. *Land*.

[23] Taghizadeh-Mehrjardi R., Nabiollahi K., Rasoli L., Kerry R., Scholten T. (2020). Land suitability assessment and agricultural production sustainability using machine learning models. *Agronomy*.

[24] Knoll L., Breuer L., Bach M. (2019). Large scale prediction of groundwater nitrate concentrations from spatial data using machine learning. *Science of the Total Environment*.

[25] Talukdar S., Singha P., Mahato S. (2020). Land-use land-cover classification by machine learning classifiers for satellite observations-A review. *Remote Sensing*.

[26] Liakos K. G., Busato P., Moshou D., Pearson S., Bochtis D. (2018). Machine learning in agriculture: a review. *Sensors*.

